The article "The Role of Adjunctive Chemical Solutions in the Treatment of Odontogenic Keratocysts: A Scoping Review" was published in 2023. Journal: Cureus.

# The Role of Adjunctive Chemical Solutions in the Treatment of Odontogenic Keratocysts: A Scoping Review

**DOI:** 10.7759/cureus.41822

**Published:** 2023-07-13

**Authors:** Munish Kumar, Arpit Tripathi, Gagandeep Singh, Amrinder Singh, Ankush Gupta, Rishabh Kasrija

**Affiliations:** 1 Department of Oral and Maxillofacial Surgery, Guru Nanak Dev Dental College & Research Institute, Sunam, IND; 2 Department of Oral and Maxillofacial Surgery, JSS Dental College, Mysuru, IND

**Keywords:** reoccurrence, enucleation, scoping review, carnoy’s solution, odontogenic keratocyst

## Abstract

Odontogenic keratocysts (OKC) are aggressive cysts with a high recurrence potential. Treating them with surgical enucleation procedures alone is associated with high recurrence rates; therefore, additional or supportive treatment approaches, such as peripheral osteotomy, cryotherapy, and chemical solutions, are warranted. The objective of the present review was to evaluate the existing literature on the efficacy of chemical approaches, such as Carnoy’s solution (CS), in preventing recurrence after the enucleation of OKC. An electronic search was conducted on PubMed, Scopus, and Google Scholar databases to find articles published from January 2010 to December 2022 by using the Medical Subject Headings (MeSH) terms “Odontogenic Keratocyst” “Carnoy’s Solution,” “Treatment,” and “Enucleation.” Articles published in the English language were selected for the study. The PICOS criteria (population: patients with non-syndromic OKC with histopathological diagnosis and a minimum follow-up of six months; intervention and comparison: enucleation followed by adjunctive chemical therapy and standard procedure; outcome: recurrence rates; study design: retrospective and prospective studies, randomized controlled trials, and case series involving at least 10 cases of OKC) were employed. Studies involving syndromic (nevoid basal cell carcinoma) cases were excluded from the search. Seventeen studies fulfilled the inclusion criteria and the majority of them were retrospective studies, with a few case series. OKC was found more frequently in the mandible, with a recurrence rate of 11%, when treated with CS following enucleation after four years of follow-up. Modified Carnoy’s solution (MC) was used in two studies. The mean follow-up period was 44 months. Based on our findings, adjuvant therapy using a chemical approach following enucleation is a more effective and beneficial modality for the treatment of OKC.

## Introduction and background

Odontogenic keratocysts (OKC) originate from the dental lamina and are classified as odontogenic cysts by WHO. Although benign, owing to its aggressive nature and high recurrence potential, its classification is controversial [1]. In 2005, WHO reclassified it as an “odontogenic keratocystic tumor,” following the unearthing of the evidence of mutation in the PTCH, p53, p16, FHIT, and MCC genes [2,3,4]. The term OKC was coined by Philipsen in 1956 [5,6].

The article "The Role of Adjunctive Chemical Solutions in the Treatment of Odontogenic Keratocysts: A Scoping Review" was published in 2023. Journal: Cureus.

An OKC is a benign odontogenic cyst that can occur in any part of the jaw. The most common locations for OKC are the ramus and body of the mandible, which may or may not be associated with the impacted tooth [2,3]. OKC has a bimodal age incidence: in the early 30s or late 70s [7]. Multiple OKCs can be associated with nevoid basal cell carcinoma syndrome (NBCCS) [2]. Radiographically, OKCs are unilocular or multilocular radiolucent lesions. They have well-defined sclerotic borders and are either uniform or scalloped. OKCs are usually associated with impacted teeth, primarily the third mandibular molar [1,5,6]. Bone expansion can be observed with root resorption of teeth in the vicinity of the cyst. Although clinical, radiographic, and operative findings such as yellow-colored fluid on aspiration are suggestive of OKC, the diagnosis is confirmed by histopathological features of corrugated and four to six layers of para- or ortho-keratinized epithelium lining the lumen [1]. The subepithelial connective tissue is densely collagenized and contains daughter cells [1,6].

The aggressive potential of OK is not well understood, and the treatment approach is also a matter of debate. The surgical procedure is determined by factors such as patient age, lesion size, important vital structures in the vicinity, and recurrence potential [8]. Some patients may only require conservative treatment, while others require an aggressive approach. The traditional treatment method employed by surgeons is enucleation (removal of the whole lesion from the bone) [7]. Conservative treatments, such as marsupialization and decompression, are also used, but due to the friable lining of the cyst and the presence of daughter cells in the subepithelial area, these treatment methods alone are not adequate [4,6]. Adjunctive methods, such as peripheral osteotomy and resection, are used to treat aggressive cysts. Other adjunctive methods, including cryotherapy, Carnoy’s solution (CS), and 5% Fluorouracil (5-FU) are also used, along with enucleation [8]. The use of CS and its modifications along with enucleation has been shown to effectively reduce the recurrence rate. CS is a fixative cauterized agent used in the lesion area after enucleation. Fixatives lead to the removal of the lining epithelium, resulting in a lower recurrence rate [6].

The objective of this scoping review was to assess the efficacy of CS and its modification in reducing the recurrence rates when used as an adjunctive approach in the treatment of OKC.

The article "The Role of Adjunctive Chemical Solutions in the Treatment of Odontogenic Keratocysts: A Scoping Review" was published in 2023. Journal: Cureus.

## Review

Methodology

This study followed the Preferred Reporting Items for Systematic Reviews and Meta-Analyses for Scoping Reviews (PRISMA-ScR) [9]. The articles obtained by searching the databases were classified using the Strength of Recommendation Taxonomy (SORT) criteria [10]. Ethical committee approval was not required for the study as it was performed based on the data from online databases. Unlike systematic reviews, scoping reviews are not registered in the International Prospective Register of Systematic Reviews (PROSPERO).

Literature Search

An exhaustive digital search was performed on PubMed (Medline), Scopus, and Google Scholar databases to find articles published from January 2010 to December 2022. "Odontogenic Keratocyst,” “Keratocystic Odontogenic Tumour,” “Odontogenic Tumour,” "Carnoy's solution,” “Treatment," and "Enucleation" were the Medical Subject Headings (MeSH) terms used. The Boolean operator "AND" was used to find the most pertinent studies.

The PICOS criteria used for the search were as follows: the studies in which OKCs without basal cell nevus syndrome were present in patients, with a minimum postoperative follow-up period of six months [Population (P)]; all studies where OKCs had been treated with enucleation along with the use of CS and its modification [Intervention (I)]; studies where the comparison was made with OKCs treated with enucleation alone [Comparator (C)]; studies where recurrence rates have been seen after treatment of OKCs [Outcome (O)]; and all types of randomized controlled trials, retrospective and prospective studies, and case series containing at least 10 cases of OKCs [Study design (S)]. 

Eligibility Criteria

The inclusion criteria were as follows: prospective or retrospective clinical studies, randomized control trials, and case series, where CS and its modifications were used as adjuvant treatment for the treatment of OKC; articles published in the English language only; those published from January 2010 to December 2022; and studies having at least 10 patients with a confirmed diagnosis of OKC. Studies in languages other than English, ambiguous reporting of the treatment used, animal studies, case reports with follow-up of less than 6 months, studies with less than 10 patients, and lesions connected to NBCC syndrome were excluded from consideration. The PRISMA-ScR flow diagram of the search is shown in Figure 1.

**Figure 1:** PRISMA-ScR flow diagram depicting the literature search PRISMA-ScR: Preferred Reporting Items for Systematic Reviews and Meta-Analyses for Scoping Reviews

Study Selection

The titles and abstracts of the articles as well as the full-text publications of all potentially relevant studies were scrutinized. The eligibility assessment was performed in an unblinded, independent manner by two reviewers (MK and AT). Consensus-based decision-making was used to settle disputes between reviewers, and a third reviewer (GS) was engaged when required. Owing to the diversity of the included papers, a meta-analysis could not be performed.

The article "The Role of Adjunctive Chemical Solutions in the Treatment of Odontogenic Keratocysts: A Scoping Review" was published in 2023. Journal: Cureus.

Results

Initial electronic and manual searches using the MeSH keywords yielded 905 articles. After removing duplicates, 654 articles were selected for review by two independent reviewers; 36 articles were found to be eligible for full-text assessment, of which 19 articles were further rejected due to the non-use of CS, an insufficient follow-up period of less than 6 six months, or having fewer than 10 cases; 17 articles were ultimately included for the final analysis (Figure 1) [11-27].

Demographic Data of the Studies

The 17 studies analyzed involved a total of 1027 patients and 1079 OKCs, and 534 were treated with enucleation followed by the use of CS. Five studies with 142 OKCs used modified Carnoy’s solution (MC) [16,20,24,25,27]. Most OKCs were found in the mandible (60-70%). The mean follow-up period was 44 months. The recurrence rate was 16.5% in the first year after the surgical procedure, 13% in two years, and 25% in four years (0-25% recurrence rate from one to four-year follow-up period). Three studies did not report recurrence after the procedure [13,16,25]. The longest follow-up period was observed in a study conducted by Zhao et al. (12-180 days) [17], in which recurrence was observed in seven out of 124 OKC cases treated by enucleation and CS. The highest level of recurrence (45%) was observed in a study by Lenorova et al. [21], where five out of 11 cases treated by enucleation and CS showed recurrence after 36 months of follow-up. Recurrence was observed in 69 out of 586 treated cases (11% recurrence rate) (Table 1).

**Table 1:** Characteristics of included studies

Authors	Year	Type of study	Number of patients	Number of OKCs	Treatment	Adjunctive treatment	Site of OKCs	Number of OKCs treated with Carnoy's	Follow-up period (months)	Recurrence, %	Recurrence, n
Gosau et al. [11]	2010	Retrospective	34	36	Enucleation	Carnoy's	Maxilla: 2, mandible: 34	14	45	14.2	2
Apajalahti et al. [12]	2011	Retrospective	46	46	Enucleation	Carnoy's	Maxilla: 19, mandible: 27	46	53	39	19
Schussel et al. [13]	2011	Retrospective	24	24	Enucleation	Carnoy's	Maxilla: 8, mandible: 16	2	46	0	0
Titinchi and Nortje [14]	2012	Retrospective	106	145	Enucleation	Carnoy's	Maxilla: 36, mandible: 109	9	12	11	1
Ribeiro-Junior et al. [15]	2012	Retrospective	14	14	Enucleation	Carnoy's	Maxilla: 3, mandible: 11	22	42	4	1
Güler et al. [16]	2012	Retrospective	39	43	Enucleation	Carnoy's	Maxilla: 10, mandible: 33	10	40	0	0
						Modified Carnoy's		15	40	0	0
Zhao et al. [17]	2012	Retrospective	257	257	Enucleation	Carnoy's	Not available	124	12–180	5.6	7
Rao and Kumar [18]	2014	Retrospective	32	34	Enucleation	Carnoy's	Maxilla: 4, mandible: 30	32	32	6.3	2
Sánchez-Burgos et al. [19]	2014	Retrospective	55	55	Enucleation	Carnoy's	Maxilla: 10, mandible: 45	14	60	14	2
Dashow et al. [20]	2015	Retrospective	80	80	Enucleation	Carnoy's	Maxilla: 24, mandible: 26	44	44	10	4
						Modified Carnoy's		36	27	35	13
Levorová et al. [21]	2015	Retrospective	22	22	Enucleation	Carnoy's	Maxilla: 6, mandible: 16	11	36	45	5
Leung et al. [22]	2016	Retrospective	105	105	Enucleation	Carnoy's	Maxilla: 22, mandible: 83	105	86	11	12
Gupta et al. [23]	2016	Prospective	12	12	Enucleation	Carnoy's	Maxilla: 2, mandible: 10	3	12–18	33	1
Ledderhof et al. [24]	2017	Retrospective	32	32	Enucleation	Modified Carnoy's	Maxilla: 12, mandible: 20	21	41	19	4
Alchalabi et al. [25]	2017	Prospective	29	29	Enucleation	Modified Carnoy's	Maxilla: 8, mandible: 21	29	36–72	0	0
Ribeiro-Júnior et al. [26]	2017	Retrospective	31	34	Enucleation	Carnoy's	Maxilla: 15, mandible: 16	28	43	14	4
Donnelly et al. [27]	2021	Retrospective	77	77	Enucleation	Carnoy's	Maxilla: 23, mandible: 54	36	24	13	5
						Modified Carnoy's		41	24	14	6

Discussion

OKC is a rare, benign but aggressive odontogenic cystic lesion with a high recurrence rate. It is most commonly found in the posterior mandible, affecting the third molar and ascending ramus area, compared with the maxilla. Males are more commonly affected than females; while it is usually seen in the second-third decades of life, it can affect people of all ages [5]. OKCs are classified as unilocular or multilocular based on their radiographic appearance. There is much controversy regarding the treatment of OKC, which ranges from simple enucleation of small cysts of less than 1 cm to extensive surgical resection in cases of cysts involving most of the jaw bone segment [4,5]. Enucleation is the most commonly performed treatment for OKC. Owing to the high recurrence rate (6-24%), CS or MC, either before enucleation or after enucleation is used. Mostly, it is applied after enucleation to reduce the recurrence rate [4,6].

The article "The Role of Adjunctive Chemical Solutions in the Treatment of Odontogenic Keratocysts: A Scoping Review" was published in 2023. Journal: Cureus.

A scoping review is a relatively new approach that provides insights into the current evidence available on a particular topic. Its methodology is almost the same as that of a systematic review, but it does not provide critically appraised and synthesized results; therefore, it does not require the assessment of methodological limitations and risk of bias, unlike a systematic review [9].

In this review, we identified 17 studies that fulfilled our inclusion criteria. Except for two prospective studies [23,25], all other studies were retrospective. Out of the 1079 OKCs found in 1027 patients, 534 were treated with enucleation and CS, and 142 were treated with MC. In previous studies where CS and MC were compared to assess their effectiveness in the prevention of the recurrence of OKC, it was found that both were equally effective, with a recurrence rate of 14.6% after two years [21].

There is much controversy regarding the effectiveness of CS in preventing the recurrence of OKC due to the heterogeneity of the data in the literature. The majority of studies were retrospective in nature, with no standardization of the follow-up period. According to the study by Gosau et al., OKCs treated with enucleation with CS had a recurrence rate of 14.3%, compared to a recurrence rate of 2-58% in cases where only enucleation was performed without the use of CS [11]. However, the study had an element of bias in terms of the length of the follow-up period, which was different for two different groups. It has been observed that OKC recurrence predominantly occurred within five years post-surgery, and it was lower in the group in which enucleation was performed along with MC [28]. In our review, three studies did not report any recurrence of OKC after treatment during the follow-up period of 26-40 months [13,16,25]. MC was used by Alchalabi et al. [25], and CS was used in the other two studies [13,16]. CS is a fixative agent that penetrates into the cancellous spaces in the bone and thus devitalizes the residual tumor cells in the bone and helps in the postoperative regeneration of the bone. It is applied after enucleation for three to five minutes, to prevent damage to the inferior alveolar nerve [25].

Previous studies in the literature have shown that MC is associated with the side effect of neurosensory damage when applied for more than three minutes. As an alternative adjunctive therapy, 5-FU has been used due to reduced morbidity, negligible recurrence, and shortened operating time associated with it. Another limitation of using MC involves cortical perforation, where satellite cells remain after enucleation of OKC and could be a possible cause of recurrence. 5-FU is an antimetabolic drug, which can be used topically; it causes reduced multiplication, and apoptosis of satellite cells by affecting the dihydropyrimidine dehydrogenase (DPD) enzyme [24,29].

The studies revealed that OKCs mostly affect the posterior mandible, with minimal bucco-lingual expansion. They mainly extend along the length of the mandible in the body. OKC has a high recurrence rate, which mostly occurs within five years post-treatment. A recurrence rate of 16% has been observed in our studies after five years of follow-up. Several possible reasons have been stated for such a high recurrence rate in OKC. The major reason might be the presence of satellite cysts, which may be left out during the enucleation process. Secondly, the recurrence may be related to the presence of thin and fragile linings in large OKCs, which are more difficult to enucleate than cysts with thick walls. The left-out portions of the lining may lead to recurrence [8]. The recurrence rates are high if a cyst is removed in pieces, which is sometimes required to preserve the inferior alveolar nerve and other vital structures. Another possible reason for the recurrence of OKCs is their proliferation from the basal cells of the oral mucosa, particularly in the third molar area and ascending ramus of the mandible. Therefore, it is very important to remove the overlying mucosa and these satellite cysts completely to prevent recurrence. The recurrence rates are very high if OKC affects the posterior mandible, and if it appears in the fifth decade of life [1]. A high recurrence of OKC can be seen in nevoid basal cell carcinoma syndrome. It has been observed that syndromic keratocysts are more commonly associated with parakeratinization and satellite cysts than non-syndromic keratocysts. The difference in the recurrence rates found in the studies might be due to differences in the follow-up periods, the surgical techniques, and the experience of the surgeon, as well as the differential use of CS. Some studies have used CS before enucleation, whereas some studies have used it after enucleation.

The article "The Role of Adjunctive Chemical Solutions in the Treatment of Odontogenic Keratocysts: A Scoping Review" was published in 2023. Journal: Cureus.

Due to the limitations of the included studies as well as the differences in the number of participants and the follow-up periods, it was difficult to arrive at conclusive findings. The limitations of this scoping review include a lack of randomized control trials and a smaller number of prospective studies. Most of the studies were retrospective in design and case series. Moreover, scoping reviews cannot address individual case variations and various other factors that can affect the treatment of OKC, such as size, location, and extent of the lesion, accompanying soft tissue damage, and whether it was a primary or recurrent case. Due to the heterogeneity of data, a meta-analysis could not be performed. Well-designed RCTs with long-term follow-ups of at least five years are recommended to overcome these limitations and provide more comprehensive findings.

## Conclusions

Within the limitations of the review, it was concluded from the studies that both CS and MC are effective in reducing the recurrence rates in OKC after enucleation. As they fix and devitalize the residual tumor cells, they can also be used for conservative treatment of large cysts. 5-FU is another novel and effective chemical adjunctive treatment method for OKC, but further research is required to assess its efficacy.
